The article "Stakeholder Perceptions of Sustainable Infrastructure Project Delivery: A Comparative Analysis between Guangdong, Hong Kong, and Macao" was published in 2022. Journal: J Environ Public Health.

# Stakeholder Perceptions of Sustainable Infrastructure Project Delivery: A Comparative Analysis between Guangdong, Hong Kong, and Macao

**DOI:** 10.1155/2022/5398706

**Published:** 2022-09-30

**Authors:** Hongyang Li, Tingting Jiang, Peng Mao, Junwei Zheng, Yuan Fang, Martin Skitmore, Di Wu

**Affiliations:** ^1^Business School, Hohai University, Nanjing 211100, China; ^2^School of Civil Engineering and Transportation, South China University of Technology, Guangzhou 510641, China; ^3^State Key Laboratory of Subtropical Building Science, South China University of Technology, Guangzhou 510641, China; ^4^College of Civil Engineering, Nanjing Forestry University, Nanjing 210037, China; ^5^Faculty of Civil Engineering and Mechanics, Kunming University of Science and Technology, Kunming 650500, China; ^6^Department of Civil and Transportation Engineering, Guangdong University of Technology, Guangzhou 510006, China; ^7^University Professorial Fellow, Faculty of Society and Design, Bond University, Queensland, Australia; ^8^School of Architecture, Zhengzhou University, Zhengzhou 450001, China

## Abstract

China is experiencing the rapid development of infrastructure projects throughout the country, especially in the Guangdong-Hong Kong SAR-Macao SAR Greater Bay Area. This is placing the Chinese construction industry under tremendous pressure to transition to a sustainability orientation due to the various economic, social, and environmental challenges involved. The transition to more sustainable infrastructure projects requires the involvement of more stakeholders, while the multistakeholder context is of less importance when making project decisions, and this may create an adverse effect on the sustainability level of infrastructure projects. Based on the questionnaire data collected, this study addresses this issue by comparatively analysing stakeholder perceptions of sustainable infrastructure delivery between Guangdong province, Hong Kong SAR, and Macao SAR. Through independent sample *t*-tests, the disparity in perceptions between paired stakeholder groups in the Greater Bay Area (as a whole) is revealed. Three pairs, i.e., government department and supervising engineers, owners and designers, and supervising engineers and operators, are found to be the most conflicting, while contractors and supervising engineers are the least. Of the 18 sustainability items analysed, *shaped local identity and international reputation (SOC, social factor 8) is the most controversial, while value-for-money of the proposed project during its lifecycle (EOC, economic factor 5) and green design and construction (ENV, environmental factor 2) have the greatest consensus towards their roles in achieving project sustainability*. Significantly, different stakeholder perceptions between the three are also identified, and the contractor group is found to share the least consensus geographically, while the operators have the least conflict rating of the relevant importance of various sustainability factors. The thorough analysis of sustainability-related items of economy, society, and environment contributes to understanding the attitudes of the various stakeholder groups involved, which then helps reduce their conflicts during sustainable infrastructure delivery.

The article "Stakeholder Perceptions of Sustainable Infrastructure Project Delivery: A Comparative Analysis between Guangdong, Hong Kong, and Macao" was published in 2022. Journal: J Environ Public Health.

## 1. Introduction

The term “sustainability” has been gaining increasing recognition in recent years worldwide, and China is no exception [1, 2]. The Chinese government issued its 1994 China's Agenda 21: White Paper on China's Population, Environment, and Development in the 21^st^ Century, incorporating the sustainable development concept into national strategies two years later [3]. As a large energy consumer and carbon emitter, the construction industry is pressed for full implementation of the sustainability philosophy [4–7]. To date, many research institutes and researchers around the world have defined sustainable construction as, for example, “a pursuit to eliminate the negative impact on the built environment while enhancing the social health and economic development of the community as a whole” [8]. Accordingly, sustainable infrastructure is considered to approach development from a holistic viewpoint based on global and domestic sustainable development goals and durability and having regard to social, financial, and political issues; public health and wellbeing; and economic and environmental concerns [9]. Eid [10], on other hand, considered that the available sustainability rating tools (e.g., Comprehensive Assessment System for Built Environment Efficiency, CASBEE) might neglect the interactions and preferences of associated stakeholders. The variability of the interactions between infrastructure project stakeholders and their conflicting preferences makes project delivery more vulnerable and less sustainable, and thus, the effective and efficient sustainability evaluation of infrastructure necessarily involves considering the interactions and preferences of different project stakeholders [10]. In addition, there is a lack of a comprehensive integration of vulnerability measurements and undue focus on design alternatives and evaluations rather than community sustainability and vulnerability, together with a lack of holistic consideration of sustainability and important system details.

Meanwhile, China is experiencing the rapid development of infrastructure projects throughout the country, especially in Guangdong province, Hong Kong Special Administrative Region (SAR), and Macao Special Administrative Region (SAR) (known as the Guangdong-Hong Kong SAR-Macao SAR Greater Bay Area). The Greater Bay Area is an agglomeration of cities to strengthen international cooperation among “Belt and Road” countries and promote low-carbon, inclusive, coordinated, and sustainable development [11]. Extensive cooperation between Guangdong, Hong Kong SAR, and Macao SAR in various respects is emphasized, with infrastructure construction being the highest priority. This is placing the AEC (Architecture, Engineering, and Construction) practitioners in the region under tremendous pressure to transition to a sustainability orientation due to the various economic, social, and environmental challenges involved. The sustainability level of projects in the Greater Bay Area has sometimes been questioned by all sectors of the community, and some recent controversial cases (e.g., the Guangzhou waste-to-energy power plant project and the Guangzhou-Shenzhen-Hong Kong SAR high-speed rail project—Hong Kong SAR section) have added to their worries. For example, the Guangzhou-Shenzhen-Hong Kong SAR high-speed rail project (Hong Kong SAR section) in the year of 2009 generated much debate among different groups over sustainability issues from social, environmental, and economic perspectives, e.g., family values, environmental impact, cost-effectiveness, and value-for-money [12].

The article "Stakeholder Perceptions of Sustainable Infrastructure Project Delivery: A Comparative Analysis between Guangdong, Hong Kong, and Macao" was published in 2022. Journal: J Environ Public Health.

It seems impossible to satisfy all the associated economic, social, and environmental sustainability concerns simultaneously due to the tight budgets/schedules of contemporary projects [13]. On the other hand, most existing studies focus on only one or two dimensions of project/city sustainability instead of covering economic, social, and environmental aspects. Ng et al. [12] have identified four major groups of stakeholders with interests in infrastructure projects, i.e., the government and project initiator, affected groups, general public, and users, as well as pressure groups and regulators. The roles of different stakeholder groups and their interactions were then illustrated to facilitate consensus building during project public participation. However, the situation becomes more complicated when emphasizing sustainable items during infrastructure delivery, as more stakeholder groups are expected to be involved and more conflicting stakeholder concerns need to be balanced. As a result, the multistakeholder context is ignored to some extent when making sustainability-related decisions: these may lead to relatively low levels of creditability/acceptance regarding both the decision process and outcomes. However, this is not solely a Chinese problem since the conflicts stem from the mismatching histories, characteristics, genders, cultures, values, beliefs, and behaviours of different stakeholder groups rather than any ideological clash between East and West. As a possible starting point in response, this research is aimed at clarifying the attitudes of the various stakeholder groups involved towards the different economy-/society-/environment-related sustainability objectives. Through this, various economic, social, and environmental sustainability-related items can be prioritized regionally and from a multistakeholder perspective to facilitate harmonious project delivery. In response, this study involved a questionnaire survey of purposively selected respondents from government departments, owners, designers, contractors, supervising engineers, operators, end-users, and NGOs (nongovernmental organizations) in Guangdong province, Hong Kong SAR, and Macau SAR. Various data analysis tools were then used to examine the regional differences between the ranked sustainability concerns from the perspective of each stakeholder group and identify the disparity in (1) perceptions between paired stakeholder groups and (2) stakeholder group perceptions in the three geographical areas. A series of validation interviews were then conducted in the final research stage. Although this research was carried out based on the Chinese context and with a focus on the Guangdong-Hong Kong SAR-Macao SAR Greater Bay Area, the generality of its process/outcome was validated by the interviewees. The findings are expected to benefit both governments and practitioners of the three regional construction industries and those in other countries/regions by prioritizing the various stakeholder concerns and coping with the associated conflicts when delivering sustainable infrastructure projects.

The article "Stakeholder Perceptions of Sustainable Infrastructure Project Delivery: A Comparative Analysis between Guangdong, Hong Kong, and Macao" was published in 2022. Journal: J Environ Public Health.

## 2. Literature Review

To measure urban sustainability in Europe, Meijering et al. [14] conduct a Delphi study with the participation of 419 urban sustainability experts. Seven components are evaluated, including air quality, governance, energy consumption, noncar transportation infrastructure, green spaces, inequality, and CO_2_ emissions. However, these indicators may place much emphasis on the environmental dimension of urban sustainability, while the economic and social domains are mostly overlooked. On the other hand, Montalban-Domingo et al. [15], from an international perspective, identify social sustainability criteria in public-work procurement through the analysis of 451 tendering documents from 10 countries. Boz and El-adaway [16], however, reveal the sustainability indicators of civil infrastructure projects according to two benchmarks of *work* (e.g., vision, experience, cost, and vicinity) and *nature* (e.g., environment, land use, reuse and recycle, aesthetics, and proximity). Nevertheless, a comprehensive index system (covering economic, environmental, and social aspects) for assessing infrastructure project sustainability is still lacking.

Multicriteria decision analysis (MCDA) is widely applied in assessing the sustainability of projects/cities (e.g., [17, 18]). This approach, according to Belton and Stewart [19], can be defined as an “umbrella term” to describe a collection of formal approaches to take explicit account of multiple criteria in helping individuals or groups explore important decisions. More difficulties arise in multiple-objective decision-making due to the increased number of individuals/groups involved [20]. However, this is the case with most decisions currently made during the development of sustainable infrastructure projects, especially with the stronger desire of stakeholders (or stakeholder groups) to affect project implementation according to their own interests [21, 22]. Despite this, few studies evaluate project sustainability in the multistakeholder context, which may result in a conflict between the decision-maker(s) and other stakeholder groups due to the lack credibility of the decision process and outcomes. To manage this necessitates the stakeholder concept/engagement [23–26], and the attitudes of different groups towards various sustainability items are investigated as detailed in the following sections.

## 3. Research Process and Methods

As shown in Figure 1, the research was carried out in four stages of literature review, item selection, questionnaire survey, and interviews.

A comprehensive literature review was conducted, and various sustainability concerns were identified in the first phase. The Web of Science Core Collection is used to search the journal and conference papers, with *sustainable infrastructure*, *project delivery*, *stakeholder perceptions*, and *regional differences* as the search keywords. Government reports related to sustainable infrastructure were obtained from the official government website of Guangdong province, Hong Kong SAR, and Macao SAR. These were reviewed, and a list of items related to the sustainability of infrastructure projects was compiled according to their occurrence. The specific process of item selection is reported in Sustainability Items.

A questionnaire survey was then conducted in which the respondents ranked different factors according to their importance in sustainable project delivery. This was carried out in the three regions to reveal the perceptions of different stakeholder groups (i.e., government departments and groups of owners, designers, contractors, supervising engineers, operators, end-users, and NGOs) of the various sustainability factors involved. These major stakeholder groups were identified based on the findings of Ng et al. [12], Li et al. [27, 28], and Li et al. [29]. Given that sustainable construction is still in its infancy in the three geographical areas and there are a limited amount of local projects of this type, the respondents were chosen by purposive sampling with eligibility criteria comprising at least two years of working experience in infrastructure project delivery in Guangdong province/Hong Kong SAR/Macao SAR or have been users of infrastructure projects in the region. The respondents rated each sustainability item on a 7-point Likert scale from 1 (least important) to 7 (most important). Both Chinese and English versions were provided to facilitate their participation. Before distribution, a pilot study was organized with the involvement of 20 experts from government departments and groups of owners, designers, contractors, supervising engineers, operators, end-users, and NGOs. This helped check whether the question sets were intelligible, easy to answer, and unambiguous and helped determine the time taken to complete the questionnaire. For instance, the need for a 7-point, instead of 5-point, Likert scale was confirmed during the pilot study, given that a relatively wide variety of items was involved and more experienced respondents were targeted.

The article "Stakeholder Perceptions of Sustainable Infrastructure Project Delivery: A Comparative Analysis between Guangdong, Hong Kong, and Macao" was published in 2022. Journal: J Environ Public Health.

In the last stage, purposively selected experts were invited to validate the research findings of the previous phases. A series of interviews was carried out to help explain and confirm the validity of the survey results. The potential interviewees were expected to possess at least five years of working/research experience of infrastructure project delivery or to have been users of infrastructure projects in Guangdong province, Hong Kong SAR, or Macao SAR. As a result, a total of 15 interviews were conducted, involving representatives from government departments, owners, contractors, designers, end-users, academia, and NGOs, as detailed in Table 1. To expedite the interview process, all the interviewees were sent an advance package of information that included the purpose of the interview, some background information, instructions for the exercise, and a brief description of previous survey findings.

## 4. Findings

### 4.1. Sustainability Items

A total of 18 sustainability items of infrastructure projects were identified based on the criterion that each must appear in a minimum of 50% of the selected literature. These were then grouped into three categories of economic (ECO), environmental (ENV), and social (SOC) perspectives a shown in Table 2. In the economic domain, the relevant sustainability concerns are the adaptability of development to local changing needs (ECO1), availability of local job opportunities (ECO2), economic benefits to government and local citizens (ECO3), balanced development of different local economic activities (ECO4), and value-for-money of the proposed project during its lifecycle (ECO5). For the environmental domain, four items were considered as influencing project environmental sustainability: harmonization of the proposed project with the local natural setting (ENV1); green design and construction (ENV2); building design, in terms of aesthetics, density, height, and visual permeability (ENV3); and prevention and mitigation measures against air, water, and noise pollution (ENV4). From the social viewpoint, the factors of sustainable project delivery comprise the following: access to work and locations of activities (the degree of accessibility strongly affects an area's social development—the higher the degree of accessibility, the more socially sustainable) (SOC1); the creation of a safe, convenient, and comfortable pedestrian circulation and transport network (SOC2); the availability of amenities, community and welfare facilities, and provision of public open space (SOC3); being functional and acceptable in terms of tariffs to diversified social groups (SOC4); having unique local characteristics (SOC5); the conservation of local cultural and historical heritage (SOC6); reasonable compensation and relocation plans/strategies—abnormally high or low compensation and irrational relocation plans/strategies may lead to social disputes (SOC7); a shaped local identity and international reputation (SOC8); and effective public participation—the effectiveness of involving the public is critical to project success, as an overly lengthy participatory exercise may adversely affect the achievement of various project objectives) (SOC9) [14, 15, 30–54].

The article "Stakeholder Perceptions of Sustainable Infrastructure Project Delivery: A Comparative Analysis between Guangdong, Hong Kong, and Macao" was published in 2022. Journal: J Environ Public Health.

### 4.2. Questionnaire Analysis

A total of 782 questionnaires were dispatched, with 177 eligible responses (23%) finally received, as shown in Table 3.

Various tools were then used for analysing the questionnaire data, including the mean score ranking technique, independent sample *t*-tests, and analysis of variance (ANOVA).

#### 4.2.1. Ranking the Various Sustainability Concerns

The mean scores (MS) of each factor related to sustainable infrastructure project delivery rated by the respondents were calculated and ranked as shown in Table 4. This shows economy-related items to be the most important concerns for government departments in Guangdong province (adaptability of development to local changing needs, ECO1, mean score = 6.75), Hong Kong SAR (availability of local job opportunities, ECO2, mean score = 6.83), and Macao SAR (balanced development of different local economic activities, ECO4, mean score = 6.83). The Guangdong government departments also equally emphasize environment-related items of preventing and mitigating air, water, and noise pollution (ENV4, mean score = 6.75).

For the owners, both the Hong Kong SAR and Macao SAR respondents believe value-for-money of the proposed project during its lifecycle (ECO5) to be the greatest determinant of project sustainability (6.71 and 6.50, respectively). In addition, the owners consider the three social factors of SOC5 (unique local characteristics), SOC8 (shaped local identity and international reputation), and SOC9 (effective public participation) to have a similar influence (mean score = 6.50). The Guangdong owners and designers, however, rate ENV4 (prevention and mitigation measures against air, water, and noise pollution) the highest, with mean scores of 6.78 and 6.29, respectively. For the Hong Kong SAR and Macao SAR designers, SOC5 (unique local characteristics) receives the highest mean scores of 6.17 and 6.13, respectively, with the Macao SAR designers equally emphasizing lifecycle value-for-money (ECO5, mean score = 6.13). This follows [42], in which the economic, social, and environmental aspects of infrastructure project sustainability were allocated the weights of 0.35, 0.36, and 0.29, respectively.

ECO5 (lifecycle value-for-money) is the most important concern for both Guangdong and Macao SAR contractors, with mean scores of 6.11 and 6.00, respectively, while ENV2 (green design and construction) also heads the Guangdong as well as the Hong Kong SAR contractors' list with mean scores of 6.11 and 6.00, respectively. To some extent, the lifecycle value-for-money of the infrastructure projects directly determines project success or failure, and green design and construction have been generally recognized to be of great significance in construction engineering.

The Guangdong and Macao SAR supervising engineers' mean scores for ECO5 (lifecycle value-for-money) are both at their highest at 6.25 and 6.14, respectively—the Guangdong respondents paying equal attention to ENV4 (prevention and mitigation measures against air, water, and noise pollution). Their Hong Kong SAR counterparts, on the other hand, rank both SOC7 (reasonable compensation and relocation plan/strategy) and SOC8 (shaped local identity and international reputation) the highest, with the same mean score of 6.00.

The article "Stakeholder Perceptions of Sustainable Infrastructure Project Delivery: A Comparative Analysis between Guangdong, Hong Kong, and Macao" was published in 2022. Journal: J Environ Public Health.

The Guangdong operators rate ENV3 (building design in terms of aesthetics, density, height, and visual permeability), with a mean score of 6.83, their top choice, while both the Hong Kong SAR and Macao SAR operators and end-users consider SOC9 (effective public participation) the most important factor, with operator mean scores of 6.57 and 6.34, respectively and end-user mean scores of 6.78 and 6.86, respectively. The Guangdong end-users pay more attention to ENV4 (prevention and mitigation measures against air, water, and noise pollution) and SOC1 (access to work and locations of activities), with the same mean score of 6.75.

ENV4 (prevention and mitigation measures against air, water, and noise pollution) is also the top concern of Guangdong NGOs, with a mean score 6.83, while both Hong Kong SAR and Macao SAR NGOs rate SOC6 (conservation of local cultural and historical heritage) highly with mean scores of 6.63 and 6.50, respectively.

#### 4.2.2. Disparity of Perceptions between Paired Stakeholder Groups in the Three Geographical Areas

Independent sample *t*-tests were carried out to identify the perspectives of the various stakeholder groups in Guangdong province, Hong Kong SAR, and Macao SAR (as a whole) more clearly. The significance of any differences in the mean scores of paired groups was tested (*p* < 0.05, two-tailed). Levene's test was used to determine whether the variances between pairs of groups could be assumed equal—again with *p* < 0.05 as the cut-off value [55]. The factors with conflicting ratings are listed in Table 5.

All 28 pairs of stakeholder groups in the Bay Area have conflicting views regarding the importance of items related to infrastructure project sustainability. Three paired stakeholder groups are identified with most conflicting concerns (16 out of 18), namely, (1) the government department and supervising engineers, (2) owners and designers, and (3) supervising engineers and operators, which may be attributed to the difference of their positions during the lifecycle of infrastructure projects and their conflicts of interest. Their greatest differences occur in the factors of SOC7 (reasonable compensation and relocation plan/strategy, mean difference = 1.85455 for the government department and supervising engineers; 1.62857 for owners and designers) and SOC5 (unique local characteristics, mean difference = −1.56724 for the supervising engineers and operators). On the other hand, there is a significant disparity in perceptions between the contractors and supervising engineers for only 2 sustainability items, i.e., SOC5 (unique local characteristics, mean difference = 0.52909) and ENV4 (prevention and mitigation measures against air, water, and noise pollution, mean difference = −0.55455). This stakeholder group pair is therefore considered the least conflicting.

The article "Stakeholder Perceptions of Sustainable Infrastructure Project Delivery: A Comparative Analysis between Guangdong, Hong Kong, and Macao" was published in 2022. Journal: J Environ Public Health.

Of the 18 sustainability concerns, SOC8 (shaped local identity and international reputation) is the most controversial, with 22 stakeholder group pairs (out of 28) conflicting. Only six pairs of stakeholder groups, i.e., government department and owners, designers and contractors, designers and supervising engineers, designers and operators, contractors and supervising engineers, and end-users and NGOs, agree on its importance. Local identity and international reputation can only be shaped by the joint efforts of overall infrastructure projects. The benefits for some infrastructure project stakeholders are relatively few (and may be delayed) compared to their efforts made, making them uninfluential when shaping local identity and international reputation. As a result, conflicts can arise between different stakeholder groups. On the other hand, the least contentious are EOC5 (lifecycle value-for-money) and ENV2 (green design and construction) with only eight conflicting stakeholder group pairs, with almost all project stakeholders benefitting.

#### 4.2.3. Disparity of Stakeholder Group Perceptions for the Three Geographical Areas

Levene's test was first used to check for homogeneity with *p* < 0.05 as the cut-off value [55]. The differences in stakeholder perceptions between Guangdong province, Hong Kong SAR, and Macao SAR were then tested by one-way ANOVA.  Table 6 summarizes the significant results at the 5% level.

This shows that, for instance, the government department respondents from Guangdong province, Hong Kong SAR, and Macao SAR do not agree over SOC1 (access to work and locations of activities) and SOC5 (unique local characteristics). Likewise, the owners disagree over SOC5 (unique local characteristics), SOC9 (effective public participation), ENV3 (building design in terms of aesthetics, density, height, and visual permeability), and ENV4 (prevention and mitigation measures against air, water, and noise pollution). A similar situation occurs with the designers, contractors, supervising engineers, and operators, with controversial differences for some non-economy-related sustainability items. On the contrary, the end-users only disagree over economic considerations, namely, ECO3 (economic benefits to government and local citizens) and ECO4 (balanced development of different local economic activities). The NGOs, however, have different views on the economic, social, and environmental factors, comprising ECO1 (adaptability of development to the local changing needs), ECO3 (economic benefits to government and local citizens), ECO4 (balanced development of different local economic activities), SOC5 (unique local characteristics), ENV1 (harmonization of the proposed project with the local natural setting), and ENV4 (prevention and mitigation measures against air, water, and noise pollution).

The article "Stakeholder Perceptions of Sustainable Infrastructure Project Delivery: A Comparative Analysis between Guangdong, Hong Kong, and Macao" was published in 2022. Journal: J Environ Public Health.

### 4.3. Validation and Discussion

15 interviewees, from government departments, owners, contractors, designers, end-users, academia, and NGOs, participated in the validation stage and evaluated the research process/findings according to a 5-point Likert scale from 1 (poor) to 5 (excellent) against the criteria of novelty, practicality, robustness, and accountability from the holistic perspective [56], as well as verifying each point in more detail, as shown in Validation and Discussion. To improve the validity of the research findings, the interviewees involved in this stage had not participated in the survey. A series of prevalidation interviews was conducted with one interviewee from each of the seven stakeholder groups. Their feedback led to the change of using a 5-point, rather than 7-point, Likert scale as they believe it is much easier for them to distinguish/rate according to 5 ranks from poor to excellent. The results (Table 7) show that all items were rated above “4,” indicating the overall satisfactory performance of the research.

### 4.4. Involving Stakeholders in Sustainable Infrastructure Decision-Making/Evaluation

During the interviews, all the participants advocated the incorporation of a multistakeholder perspective during the decision-making/evaluation of sustainable infrastructure projects. As a representative of academia and NGOs stated, “it is a global phenomenon (rather than a solely Chinese one) that an overwhelming majority of sustainability-related project decisions are currently made in a multi-stakeholder context,” and “it is rather difficult to reach a consensus due to the existence of a significant divergence of views among the various stakeholder groups and even among the individuals from the same stakeholder group towards their sustainability-related concerns during infrastructure project delivery.”

### 4.5. The 18 Sustainability-Related Concerns and Their Rankings in the Three Geographical Areas

The 18 sustainability-related concerns of the various stakeholder groups were considered by the validation panel as comprehensively covering the economic-environmental-social aspects. Moreover, these items are consistent across the globe, even if contextual differences may dictate differences in the priority levels attached to them.

From the perspective of each stakeholder group, it is unsurprising that the government department respondents from all three regions emphasize economic sustainability concerns the most (ECO1 for Guangdong province, ECO2 for Hong Kong SAR, and ECO4 for Macao SAR). Li et al. [8] prioritized performance indicators for sustainable construction and development of education infrastructure in Australia. Their rankings coincide with the findings of this research, with the economic sustainability items most important followed by the environmental and social factors. All the validation interviewees understand such views of governments at various levels and that economic sustainability needs to be achieved without sacrificing social-environmental harmony. One Mainland China government department representative pointed out that such issues as environmental protection are increasingly emphasized, especially by the authority involved. Guangdong province is one of the largest economies in China [57], but its economic development has tended to take precedence over environmental protection [58]. As a result, the public's environmental awareness has been increasing recently [59, 60], and most Guangdong province stakeholder groups attach more importance to environment-related sustainability factors. This corresponds with the survey results, in that ENV4 (prevention and mitigation measures against air, water, and noise pollution) is paid equal attention by the government respondents from the Guangdong province. Similarly, the other stakeholder groups from Guangdong province all consider environmental items to be the most important, i.e., owners (ENV4), designers (ENV4), contractors (ENV2), supervising engineers (ENV4), operators (ENV3), end-users (ENV4), and NGOs (ENV4). The NGO interviewees added that

all the parties involved in infrastructure project delivery have shifted their awareness of environmental sustainability and our role of promoting sustainable development of this type should be strengthened especially in mainland China.

The article "Stakeholder Perceptions of Sustainable Infrastructure Project Delivery: A Comparative Analysis between Guangdong, Hong Kong, and Macao" was published in 2022. Journal: J Environ Public Health.

Most of the Macao SAR stakeholder groups, on the other hand, focus more on economy-related sustainability factors, e.g., ECO4 (balanced development of different local economic activities) for government department respondents and ECO5 (lifecycle value-for-money) for owners, designers, contractors, and supervising engineers. This indicates that, by taking into account the current economic-social-environmental situation of Macao SAR, its booming economy is the leading driver in many sectors, including the construction industry [61, 62]. The economy of Macao SAR has for a long time been overwhelmingly dependent on its gambling [63, 64] and marine industries [65]. To keep its economy developing more sustainably, it may focus more on economy-related sustainability factors for sustainable infrastructure project delivery. A Macao SAR end-user, during the validation interviewees, also suggested that some social sustainability issues should not be ignored, such as the conservation of local cultural and historical heritage (SOC6) and effective public participation (SOC9), to ensure the local economy develops in the sustainable manner.

Meanwhile, the survey revealed that the Hong Kong SAR stakeholder groups hold rather different views regarding the most important factor involved. While the government department respondents (ECO2) and owners (ECO5) pay more attention to economy-related sustainability issues, the contractors rate ENV2 the most important. The others, i.e., designers (SOC5), supervising engineers (SOC7 and SOC8), operators (SOC9), end-users (SOC9), and NGOs (SOC6), all consider social sustainability to overshadow economic and environmental sustainability. Hong Kong SAR is a global financial centre [66], and thus, the government department respondents and owners may place a greater emphasis on economy-related sustainability items to maintain social stability. Population's high density is one of its most serious restraints on sustainable development [67]. With such a large population being affected, society-related sustainability issues must be taken into consideration in the delivery of infrastructure projects. The academic and end-user validation interviewees further explained that social issues have become the main barrier hindering the development of Hong Kong SAR and that

due to the project nature, infrastructure delivery has always been the focus of the whole society. As a result, some social sustainability-related concerns should be preferentially satisfied when developing projects of this type.

### 4.6. Comparison of Perceptions of Stakeholder Groups in the Three Geographical Areas

From the perspective of the paired stakeholder groups in the three regions, the most conflicting pairs (disagreeing over 16 sustainability objectives) are (1) the government department respondents and supervising engineers, (2) owners and designers, and (3) supervising engineers and operators. These three most conflicting pairs comprise stakeholders in different stages of the infrastructure project lifecycle: government department respondents and designers for the design stage, supervising engineers for the construction stage, and the owners and operators who may focus more on the operation stage. Their benefits when delivering infrastructure projects are often conflicting, and thus, their attitudes towards these 18 sustainability items tend to be quite diverse. Conversely, the contractors and supervising engineers agree on 16 items. The designers and contractors have a total of 80 conflicts with the other stakeholder groups, while NGOs have 63 conflicts with government department respondents, owners, designers, contractors, supervising engineers, operators, and end-users. During the validation interviews, the designers and contractors pointed out that it is rather difficult to balance economic, social, and environmental sustainability during the design and construction stages, stating that “simultaneously satisfying owners and end-users seems a mission impossible for us.”

The article "Stakeholder Perceptions of Sustainable Infrastructure Project Delivery: A Comparative Analysis between Guangdong, Hong Kong, and Macao" was published in 2022. Journal: J Environ Public Health.

SOC8 (shaped local identity and international reputation) is the most controversial of the sustainability factors, with 22 (out of 28) conflicting stakeholder group pairs, while EOC5 (lifecycle value-for-money) and ENV2 (green design and construction) are the least, with only 8 conflicting pairs. In response, the Mainland China government representatives deem it inappropriate to gain international reputation at the cost of losing local identity, implying the need for Chinese people to be more confident of their cultural characteristics.

Regionally, the contractors have the most conflicting sustainability concerns (7 out of 18). The respondents from Guangdong, Hong Kong SAR, and Macao SAR agree on the importance of all the economy-related sustainability factors, but with disparate perceptions of SOC1 (access to work and locations of activities), SOC2 (creation of a safe, convenient, comfortable, and legible pedestrian circulation and transport network), SOC5 (unique local characteristics), SOC8 (shaped local identity and international reputation), ENV1 (harmonization with the local natural setting), ENV3 (building design in terms of aesthetics, density, height, and visual permeability), and ENV4 (prevention and mitigation measures against air, water, and noise pollution). Of these, the greatest difference is in SOC5 (*F* = 17.453). Three academic representatives from Guangdong, Hong Kong SAR, and Macao SAR explained that, compared with the China mainland, Hong Kong SAR practitioners place a greater emphasis on maintaining unique local characteristics, while it seems that the mainland may have taken an early wrong path by simply copying some single modes when developing new projects/areas. Today, Mainland China practitioners are increasingly realizing the importance of retaining local features. As a result, the Chinese style is expected to be further promoted while gaining a global reputation from a shaped local identity.

## 5. Conclusions

This study focuses on stakeholder perceptions of sustainable infrastructure project delivery in the Chinese regions of Guangdong province, Hong Kong SAR, and Macao SAR. A total of 18 sustainability considerations (with 5, 4, and 9 items from economic, environmental, and social domains, respectively) were derived from a global literature review and then rated/ranked in terms of their importance in delivering sustainable infrastructure projects by government departments, owners, designers, contractors, supervising engineers, operators, end-users, and NGOs in the three geographical areas through a survey. Regional disparities in perceptions between paired stakeholder groups were later revealed by independent sample *t*-tests. The results indicate the most conflicting stakeholder group pairs to be (1) government department respondents and supervising engineers, (2) owners and designers, and (3) supervising engineers and operators, while the least conflicting are contractors and supervising engineers. On the other hand, the most controversial sustainability factor is SOC8 (shaped local identity and international reputation), while EOC5 (lifecycle value-for-money) and ENV2 (green design and construction) are the least contentious. The different stakeholder perceptions among the three geographical areas are also identified through one-way ANOVA, with the contractor group emerging as the most conflicting in all the three regions. The operators, on the other hand, share similar views concerning most of the economic, social, and environmental sustainability items. These provide the basis for prioritizing various stakeholder relationships/concerns during the delivery of sustainable projects in the future.

The article "Stakeholder Perceptions of Sustainable Infrastructure Project Delivery: A Comparative Analysis between Guangdong, Hong Kong, and Macao" was published in 2022. Journal: J Environ Public Health.

For the theoretical implications, participative decision-making/evaluation is a potential solution to help achieve project sustainability objectives. As a result, stakeholders are emphasized throughout this research, and their participation during the project lifecycle is encouraged to help solve conflicts and reach a consensus. Through this, infrastructure projects are expected to be delivered in a smooth and sustainable manner. Theoretically, this study specifically applies MCDA to sustainable infrastructure project delivery from a multistakeholder perspective, which helps broaden the application of MCDA theory. From a more practically perspective, specific strategies are provided to facilitate the development of sustainable infrastructure projects in the Guangdong-Hong Kong SAR-Macao SAR Greater Bay Area. These include the following: (1) more attention needs to be paid to improving the environmental (for Guangdong), social (for Hong Kong SAR), and economic (for Macao SAR) sustainability levels when delivering infrastructure projects in the three regions; (2) channels should be established between various stakeholder groups (especially between government departments and supervising engineers, owners and designers, and supervising engineers and operators) to maintain their dialogues in a respectful and inclusive way; (3) the sustainability factor of shaped local identity and international reputation should be treated carefully in the Bay Area to avoid potential conflicts; and (4) the participation of contractors should be enhanced during sustainable infrastructure project delivery. The research findings are valuable for the AEC industries of both the Guangdong-Hong Kong SAR-Macao SAR Greater Bay Area and other countries/regions when managing stakeholders, building a consensus (for the Guangdong-Hong Kong SAR-Macao SAR Greater Bay Area—especially between the most conflicting stakeholder group pairs as revealed from the survey analysis, e.g., government departments and supervising engineers, owners and designers, and supervising engineers and operators), and facilitating the smooth delivery of sustainable infrastructure projects.

The article "Stakeholder Perceptions of Sustainable Infrastructure Project Delivery: A Comparative Analysis between Guangdong, Hong Kong, and Macao" was published in 2022. Journal: J Environ Public Health.

The study is limited by the validation results in Validation and Discussion and Table 7 being concerned with the research findings as a whole—the detailed correlation with each sustainability item needs to be examined in the future. More validation interviewees should be invited in the future to ensure the stakeholder representativeness in each geographical area. Moreover, while the Guangdong-Hong Kong SAR-Macao SAR Greater Bay Area is used to analyse stakeholder perceptions of sustainable infrastructure delivery, the extent to which the findings of this research apply outside of the Chinese context is a topic for further study. Future studies will also benefit from carrying out comparative studies between China and other countries/regions regarding stakeholder management theory/practice when delivering sustainable infrastructure projects of different types (e.g., civil construction, roads, bridges, schools, and parks). In addition, since the study was conducted in 2018, the COVID-19 pandemic is not considered and its impact on the stakeholders' perception of the sustainability in the architecture, engineering, and construction is worthy of in-depth study. Furthermore, more detailed measures should be investigated to facilitate the development of sustainable infrastructure projects.

## Figures and Tables

**Figure 1:** Research workflow.

**Table 1:** Interviewee profiles during validation.

Group	No.	Region	Position	Organization
Government department	1	Guangdong province	Deputy director	Municipal bureau
	2	Macao SAR	Director	Government department
Owner	3	Hong Kong SAR	Project manager	Real estate corporation
	4	Macao SAR	General manager	Real estate corporation
Contractor	5	Guangdong province	Engineer	Construction company
	6	Hong Kong SAR	Deputy manager	Construction company
Designer	7	Guangdong province	Manager	Design company
	8	Hong Kong SAR	Architect	Design consultants
End-user	9	Macao SAR	End-user	N/A
	10	Hong Kong SAR	End-user	N/A
Academia	11	Hong Kong SAR	Associate professor	University
	12	Guangdong province	Research fellow	Municipal research institution
	13	Macao SAR	Associate professor	University
NGOs	14	Guangdong province	Member	NGO
	15	Hong Kong SAR	Member	NGO

The article "Stakeholder Perceptions of Sustainable Infrastructure Project Delivery: A Comparative Analysis between Guangdong, Hong Kong, and Macao" was published in 2022. Journal: J Environ Public Health.

**Table 2:** Sustainability items of infrastructure projects.

Sustainability items of infrastructure projects		
Economic (ECO) domain	Environmental (ENV) domain	Social (SOC) domain
(1) Adaptability of development to local changing needs (ECO1) (FA = 81%)	(1) Harmonization of the proposed project with the local natural setting (ENV1) (FA = 70%)	(1) Access to work and locations of activities (SOC1) (FA = 78%)
(2) Availability of local job opportunities (ECO2) (FA = 63%)	(2) Green design and construction (ENV2) (FA = 81%)	(2) Creation of a safe, convenient, comfortable, and legible pedestrian circulation and transport network (SOC2) (FA = 78%)
(3) Economic benefits to government and local citizens (ECO3) (FA = 78%)	(3) Building design in terms of aesthetics, density, height, and visual permeability (ENV3) (FA = 74%)	(3) Availability of amenities, community and welfare facilities, and provision of public open space (SOC3) (FA = 74%)
(4) Balanced development of different local economic activities (ECO4) (FA = 78%)	(4) Prevention and mitigation measures against air, water, and noise pollution (ENV4) (FA = 70%)	(4) Being functional and acceptable in terms of tariffs to diversified social groups (SOC4) (FA = 59%)
(5) Value-for-money of the proposed project during its lifecycle (ECO5) (FA = 67%)		(5) Unique local characteristics (SOC5) (FA = 74%)
		(6) Conservation of local cultural and historical heritage (SOC6) (FA = 63%) (7) Reasonable compensation and relocation plans/strategies (SOC7), (FA = 63%) (8) Shaped local identity and international reputation (SOC8) (FA = 74%) (9) Effective public participation (SOC9) (FA = 70%)

FA denotes the frequency of appearance of a certain item in the selected literature.

**Table 3:** Response rate of the questionnaire survey conducted in this research.

	Government department	Owners	Designers	Contractors	Supervising engineers	Operators	End-users	NGOs	Overall
*Guangdong province*									
Distributed	34	35	32	39	37	29	35	27	268
Received	8	10	7	9	8	6	8	6	62
Response rate	24%	29%	22%	23%	22%	27%	23%	22%	23%

*Hong Kong SAR*									
Distributed	28	33	29	35	31	32	36	34	258
Received	6	7	6	7	7	7	9	8	57
Response rate	21%	21%	21%	20%	23%	22%	25%	24%	22%

*Macao SAR*									
Distributed	30	36	32	40	28	30	30	30	256
Received	6	8	8	9	7	7	7	6	58
Response rate	20%	22%	25%	23%	25%	23%	23%	20%	23%

*Total*									
Distributed	92	104	93	114	96	91	101	91	782
Received	20	25	21	25	22	20	24	20	177
Response rate	22%	24%	23%	22%	23%	22%	24%	22%	23%

**(a):** 

Sustainability concern	Stakeholder groups																							
	Government department			Owners			Designers			Contractors			Supervising engineers			Operators			End-users			NGOs		
	GD	HK	MC	GD	HK	MC	GD	HK	MC	GD	HK	MC	GD	HK	MC	GD	HK	MC	GD	HK	MC	GD	HK	MC
ECO1	6.75 (1)	6.67 (2)	6.50 (3)	5.70 (11)	6.14 (9)	6.13 (10)	5.14 (12)	4.67 (17)	5.25 (9)	5.33 (8)	4.71 (13)	5.22 (9)	5.38 (9)	5.29 (9)	5.43 (8)	6.00 (9)	5.43 (15)	5.86 (13)	5.88 (15)	5.33 (16)	6.00 (13)	6.50 (2)	5.38 (14)	6.33 (2)
ECO2	6.63 (3)	6.83 (1)	6.67 (2)	5.80 (9)	6.00 (13)	6.00 (15)	5.00 (13)	5.67 (3)	5.13 (10)	5.78 (5)	5.86 (2)	5.89 (2)	5.63 (5)	5.86 (3)	5.86 (2)	6.17 (6)	6.00 (9)	6.29 (2)	6.38 (9)	5.78 (15)	6.43 (4)	5.83 (12)	5.25 (15)	6.00 (8)
ECO3	6.50 (4)	6.67 (2)	6.50 (3)	5.60 (13)	5.86 (16)	6.13 (10)	5.43 (8)	5.33 (8)	5.50 (4)	5.44 (7)	4.86 (11)	5.67 (5)	5.50 (8)	5.71 (7)	5.57 (6)	6.00 (9)	6.00 (9)	6.14 (9)	6.63 (3)	5.89 (13)	6.57 (2)	6.00 (11)	4.75 (16)	6.17 (5)
ECO4	6.38 (7)	6.50 (5)	6.83 (1)	5.50 (14)	6.00 (13)	6.25 (6)	5.00 (13)	4.33 (18)	5.13 (10)	4.89 (11)	4.57 (14)	4.78 (14)	5.00 (12)	5.00 (15)	5.00 (14)	5.83 (15)	5.14 (18)	5.86 (13)	6.13 (12)	5.33 (16)	6.14 (11)	6.17 (9)	4.63 (17)	6.00 (8)
ECO5	6.00 (14)	6.33 (9)	6.33 (8)	6.60 (2)	6.71 (1)	6.50 (1)	6.00 (2)	5.50 (5)	6.13 (1)	6.11 (1)	5.43 (6)	6.00 (1)	6.25 (1)	5.86 (3)	6.14 (1)	6.17 (6)	6.14 (6)	6.14 (9)	6.00 (13)	6.00 (11)	5.86 (15)	6.33 (7)	6.00 (10)	6.17 (5)
ENV1	6.13 (12)	5.67 (17)	5.67 (17)	6.00 (7)	6.14 (9)	6.13 (10)	5.86 (4)	5.17 (11)	5.00 (13)	5.78 (5)	4.43 (18)	4.33 (18)	5.75 (4)	4.43 (18)	4.29 (18)	6.67 (2)	5.43 (15)	5.29 (18)	6.50 (7)	6.11 (9)	5.86 (15)	6.33 (7)	5.63 (12)	5.50 (16)
ENV2	6.50 (4)	6.50 (5)	6.33 (8)	6.10 (5)	6.29 (6)	6.13 (10)	6.00 (2)	5.83 (2)	5.38 (8)	6.11 (1)	6.00 (1)	5.67 (5)	5.88 (3)	5.86 (3)	5.71 (4)	6.50 (4)	5.86 (12)	5.71 (17)	6.25 (11)	6.11 (9)	5.86 (15)	6.50 (2)	6.25 (5)	6.00 (8)
ENV3	6.25 (9)	6.00 (15)	5.83 (15)	6.30 (3)	6.29 (6)	5.75 (17)	5.71 (5)	5.33 (8)	5.00 (13)	5.89 (4)	5.29 (8)	5.22 (9)	5.63 (5)	5.14 (13)	5.00 (14)	6.83 (1)	6.29 (3)	6.14 (9)	6.63 (3)	6.44 (4)	6.43 (4)	6.50 (2)	6.13 (7)	5.67 (15)
ENV4	6.75 (1)	6.33 (9)	6.00 (13)	6.78 (1)	5.86 (16)	6.00 (15)	6.29 (1)	4.83 (14)	4.75 (18)	6.00 (3)	5.14 (9)	5.00 (12)	6.25 (1)	5.86 (3)	5.71 (4)	6.67 (2)	6.43 (2)	6.29 (2)	6.75 (1)	6.44 (4)	6.29 (7)	6.83 (1)	6.38 (2)	6.00 (8)

Note: GD: Guangdong province; HK: Hong Kong SAR; and MC: Macao SAR. *N* denotes the ranking of a sustainability concern among the overall 18 items as rated by a stakeholder group in a region (*N* ∈ 1 ~ 18).

**(b):** 

Sustainability concern	Stakeholder groups																							
	Government department			Owners			Designers			Contractors			Supervising engineers			Operators			End-users			NGOs		
	GD	HK	MC	GD	HK	MC	GD	HK	MC	GD	HK	MC	GD	HK	MC	GD	HK	MC	GD	HK	MC	GD	HK	MC
SOC1	4.88 (17)	6.00 (15)	5.83 (15)	6.10 (5)	6.14 (9)	6.25 (6)	4.86 (15)	5.33 (8)	5.50 (4)	4.67 (13)	5.71 (4)	5.78 (3)	4.38 (14)	5.29 (9)	5.43 (8)	6.33 (5)	6.14 (6)	6.21 (5)	6.75 (1)	6.44 (4)	6.29 (7)	5.83 (12)	5.50 (13)	5.33 (17)
SOC2	6.13 (12)	5.67 (17)	5.67 (17)	5.80 (9)	6.29 (6)	6.25 (6)	5.29 (9)	4.83 (14)	4.88 (16)	5.33 (8)	4.57 (14)	4.67 (15)	5.25 (10)	4.71 (17)	4.86 (16)	6.17 (6)	5.86 (12)	5.83 (13)	6.63 (3)	6.33 (7)	6.29 (7)	6.17 (9)	5.88 (11)	5.83 (14)
SOC3	6.00 (14)	6.50 (5)	6.17 (12)	5.70 (11)	6.14 (9)	6.25 (6)	5.57 (7)	5.50 (5)	5.50 (4)	4.67 (13)	5.00 (10)	5.11 (11)	4.50 (13)	5.29 (9)	5.43 (8)	6.00 (9)	6.14 (6)	6.21 (5)	6.38 (9)	6.67 (2)	6.57 (2)	5.67 (15)	6.38 (2)	6.33 (2)
SOC4	5.63 (16)	6.17 (14)	6.33 (8)	5.50 (14)	6.00 (13)	6.13 (10)	4.29 (17)	4.83 (14)	4.88 (16)	4.44 (15)	4.57 (14)	4.67 (15)	4.00 (15)	5.14 (13)	5.29 (12)	6.00 (9)	6.29 (3)	6.17 (7)	6.50 (7)	6.56 (3)	6.43 (4)	5.33 (16)	6.13 (7)	6.00 (8)
SOC5	4.88 (17)	6.33 (9)	6.00 (13)	4.40 (18)	6.57 (2)	6.50 (1)	5.29 (9)	6.17 (1)	6.13 (1)	4.22 (17)	5.71 (4)	5.56 (7)	3.88 (17)	4.86 (16)	5.14 (13)	6.00 (9)	6.29 (3)	6.17 (7)	6.00 (13)	5.89 (13)	6.00 (13)	5.17 (17)	6.13 (7)	6.17 (5)
SOC6	6.25 (9)	6.50 (5)	6.50 (3)	5.30 (17)	5.71 (18)	5.75 (17)	5.29 (9)	5.17 (11)	5.13 (10)	4.78 (12)	5.43 (6)	5.44 (8)	5.63 (5)	5.43 (8)	5.57 (6)	5.67 (17)	6.00 (9)	6.24 (4)	5.25 (17)	6.00 (11)	6.14 (11)	6.50 (2)	6.63 (1)	6.50 (1)
SOC7	6.50 (4)	6.33 (9)	6.33 (8)	5.90 (8)	6.43 (3)	6.38 (5)	3.71 (18)	5.00 (13)	5.00 (13)	4.11 (18)	4.57 (14)	4.56 (17)	3.88 (17)	6.00 (1)	4.86 (16)	5.17 (18)	5.43 (15)	5.86 (13)	5.88 (15)	6.33 (7)	6.29 (7)	5.83 (12)	6.25 (5)	6.00 (8)
SOC8	6.38 (7)	6.67 (2)	6.50 (3)	6.20 (4)	6.43 (3)	6.50 (1)	5.71 (5)	5.67 (3)	5.50 (4)	4.33 (16)	5.86 (2)	5.78 (3)	4.00 (16)	6.00 (1)	5.86 (2)	6.00 (9)	5.86 (12)	5.98 (12)	4.63 (18)	4.33 (18)	4.43 (18)	3.83 (18)	4.25 (18)	4.33 (18)
SOC9	6.25 (9)	6.33 (9)	6.50 (3)	5.50 (14)	6.43 (3)	6.50 (1)	4.86 (15)	5.50 (5)	5.63 (3)	5.11 (10)	4.86 (11)	4.89 (13)	5.13 (11)	5.29 (9)	5.43 (8)	5.83 (15)	6.57 (1)	6.34 (1)	6.63 (3)	6.78 (1)	6.86 (1)	6.50 (2)	6.38 (2)	6.33 (2)

Note: GD: Guangdong province; HK: Hong Kong SAR; and MC: Macao SAR. *N* denotes the ranking of a sustainability concern among the overall 18 items as rated by a stakeholder group in a region (*N* ∈ 1 ~ 18).

**(a):** 

Items related to infrastructure project sustainability																			
Paired stakeholder groups	ECO1	ECO2	ECO3	ECO4	ECO5	SOC1	SOC2	SOC3	SOC4	SOC5	SOC6	SOC7	SOC8	SOC9	ENV1	ENV2	ENV3	ENV4	Sum
Government department vs. owners	√	√	√	√	√	√					√								7
Government department vs. designers	√	√	√	√			√	√	√		√	√	√	√	√	√	√	√	15
Government department vs. contractors	√	√	√	√			√	√	√		√	√	√	√	√	√	√	√	15
Government department vs. supervising engineers	√	√	√	√			√	√	√	√	√	√	√	√	√	√	√	√	16
Government department vs. operators	√	√	√	√		√				√	√	√	√			√			10
Government department vs. end-users	√	√		√		√	√		√		√		√	√		√	√		11
Government department vs. NGOs	√	√	√	√									√						5
Owners vs. designers	√	√	√	√	√	√	√	√	√			√	√	√	√	√	√	√	16
Owners vs. contractors	√		√	√	√	√	√	√	√			√	√	√	√		√	√	14
Owners vs. supervising engineers	√			√	√	√	√	√	√	√		√	√	√	√		√		13

**(b):** 

Items related to infrastructure project sustainability																			
Paired stakeholder groups	ECO1	ECO2	ECO3	ECO4	ECO5	SOC1	SOC2	SOC3	SOC4	SOC5	SOC6	SOC7	SOC8	SOC9	ENV1	ENV2	ENV3	ENV4	Sum
Owners vs. operators					√						√	√	√						4
Owners vs. end-users			√		√			√	√				√	√			√		7
Owners vs. NGOs					√	√					√		√						4
Designers vs. contractors		√						√		√				√					4
Designers vs. supervising engineers		√						√		√								√	4
Designers vs. operators	√	√	√	√		√	√	√	√		√	√		√			√	√	13
Designers vs. end-users	√	√	√	√		√	√	√	√		√	√	√	√	√		√	√	15
Designers vs. NGOs	√			√			√	√	√		√	√	√	√	√	√	√	√	13
Contractors vs. supervising engineers										√								√	2
Contractors vs. operators	√		√	√		√	√	√	√	√	√	√	√	√	√		√	√	15

**(c):** 

Items related to infrastructure project sustainability																			
Paired stakeholder groups	ECO1	ECO2	ECO3	ECO4	ECO5	SOC1	SOC2	SOC3	SOC4	SOC5	SOC6	SOC7	SOC8	SOC9	ENV1	ENV2	ENV3	ENV4	Sum
Contractors vs. end-users	√		√	√		√	√	√	√	√	√	√	√	√	√		√	√	15
Contractors vs. NGOs	√			√			√	√	√	√	√	√	√	√	√		√	√	13
Supervising engineers vs. operators	√	√	√	√		√	√	√	√	√	√	√	√	√	√		√	√	16
Supervising engineers vs. end-users		√	√	√	√	√	√	√	√	√		√	√	√	√		√	√	15
Supervising engineers vs. NGOs	√					√	√	√	√	√	√	√	√	√	√	√	√	√	14
Operators vs. end-users							√	√				√	√	√					5
Operators vs. NGOs		√				√					√	√	√						5
End-users vs. NGOs		√	√			√	√	√	√		√			√			√		9
Overall	18	16	16	18	8	16	18	20	18	12	18	19	22	20	14	8	18	16	295

The article "Stakeholder Perceptions of Sustainable Infrastructure Project Delivery: A Comparative Analysis between Guangdong, Hong Kong, and Macao" was published in 2022. Journal: J Environ Public Health.

**Table 6:** Significantly different regional stakeholder perceptions.

Stakeholder groups	Stakeholder perceptions with significant difference	Sum of squares	df	Mean square	*F*	Sig.
Government department	SOC1 (between groups)	5.292	2	2.646	5.835	.012
	SOC5 (between groups)	8.342	2	4.171	8.638	.003

Owners	SOC5 (between groups)	27.326	2	13.663	37.044	.000
	SOC9 (between groups)	5.626	2	2.813	6.058	.008
	ENV3 (between groups)	1.611	2	.806	3.525	.047
	ENV4 (between groups)	4.583	2	2.291	7.807	.003

Designers	SOC5 (between groups)	3.435	2	1.717	9.854	.001
	SOC7 (between groups)	7.714	2	3.857	7.364	.005
	ENV1 (between groups)	2.976	2	1.488	4.707	.023
	ENV4 (between groups)	10.524	2	5.262	25.177	.000

Contractors	SOC1 (between groups)	6.776	2	3.388	8.296	.002
	SOC2 (between groups)	2.926	2	1.463	4.172	.029
	SOC5 (between groups)	11.434	2	5.717	17.453	.000
	SOC8 (between groups)	12.627	2	6.314	11.190	.000
	ENV1 (between groups)	11.370	2	5.685	17.204	.000
	ENV3 (between groups)	2.367	2	1.183	4.433	.024
	ENV4 (between groups)	5.143	2	2.571	5.211	.014

Supervising engineers	SOC1 (between groups)	4.982	2	2.491	4.296	.029
	SOC3 (between groups)	3.812	2	1.906	7.041	.005
	SOC4 (between groups)	7.578	2	3.789	8.688	.002
	SOC5 (between groups)	6.729	2	3.364	13.929	.000
	SOC8 (between groups)	19.006	2	9.503	14.044	.000
	ENV1 (between groups)	9.948	2	4.974	14.227	.000

Operators	ENV1 (between groups)	7.274	2	3.637	7.294	.005

End-users	ECO3 (between groups)	2.855	2	1.428	3.536	.047
	ECO4 (between groups)	3.601	2	1.801	4.890	.018

NGOs	ECO1 (between groups)	5.292	2	2.646	6.705	.007
	ECO3 (between groups)	8.617	2	4.308	16.902	.000
	ECO4 (between groups)	10.292	2	5.146	13.040	.000
	SOC5 (between groups)	4.008	2	2.004	7.502	.005
	ENV1 (between groups)	2.492	2	1.246	4.498	.027
	ENV4 (between groups)	2.092	2	1.046	3.776	.044

**Table 7:** Validation results.

Group	No.	Validation criteria			
		Novelty	Practicality	Robustness	Accountability
Government department	1	5	4	5	5
	2	4	4	5	5
Owner	3	4	5	5	4
	4	5	5	4	5
Contractor	5	5	5	5	5
	6	5	3	4	4
Designer	7	4	4	4	5
	8	4	4	5	5
End-user	9	5	5	4	5
	10	5	4	5	4
Academia	11	5	5	5	5
	12	4	5	4	5
	13	5	4	4	5
NGOs	14	5	5	5	4
	15	4	5	4	4
Mean		4.60	4.47	4.53	4.67

## Data Availability

The data used to support the findings of this study are available from the corresponding author upon request.
